RETRACTED

# Judgement of the Clinical Value of Spiral CT Three-Dimensional Reconstruction in the Diagnosis of Lumbar Degenerative Osteoporosis

**DOI:** 10.1155/2022/3527156

**Published:** 2022-02-22

**Authors:** Zhe Li, Zhi Qing Ju, Tian Cheng Wang, Li Li Xin

**Affiliations:** ^1^Department of Spinal Surgery, The Affiliated Hospital of Chengde Medical College, Chengde, 067000 Hebei, China; ^2^Department of Rehabilitation, The Affiliated Hospital of Chengde Medical College, Chengde, 067000 Hebei, China; ^3^Department of Endocrinology, The Affiliated Hospital of Chengde Medical College, Chengde, 067000 Hebei, China

## Abstract

With the aging of the population, there are more and more degenerative diseases of the lumbar spine that accompany osteoporosis. Lumbar degenerative osteoporosis has also become fragile and high in incidence, which has also attracted the attention of experts and scientists in related fields. Degeneration of the lumbar spine often causes pain in the waist and surrounding patients and even affects their life safety. The lesions such as the shoulders and lower back often show varying degrees of softening or induration in the fracture line or osteoporosis will directly produce adverse reactions to joint activities and then cause the development and deterioration of various complications. At present, spiral CT three-dimensional reconstruction technology has been widely used in the field of medical imaging and has played a very important role in the diagnosis and treatment of some diseases. Therefore, combined with three-dimensional reconstruction of spiral CT, this paper discusses its clinical value in the diagnosis of lumbar degenerative osteoporosis. In this experiment, in order to understand the image results after three-dimensional reconstruction, five groups of cases were selected for testing. The test items include the whole lesion site, vertebral imaging, soft tissue lesion site, and lumbar lesion site. In addition, in order to understand the clinical value of spiral CT three-dimensional reconstruction in the diagnosis of lumbar degenerative osteoporosis, this technique was compared and tested with other imaging methods. The selected imaging methods include X-ray, CT, and MRI. The test items include sensitivity, accuracy, positive predictive value, and negative predictive value. To explore the clinical value of spiral CT three-dimensional reconstruction in the diagnosis of lumbar degenerative osteoporosis, from the experimental results, the relevant image clarity and accuracy of the five groups of cases are high, the image quality after three-dimensional reconstruction is good, and the clarity and accuracy are high. In addition, the sensitivity and accuracy of spiral CT three-dimensional reconstruction are higher than those of other imaging methods. It has great clinical value in the diagnosis and treatment of lumbar degenerative osteoporosis.

RETRACTED

## 1. Introduction

At present, osteoporosis is more common in the elderly, but now it is gradually approaching the younger population. Studies have shown that the occurrence of osteoporosis is often accompanied by degenerative lesions of the lumbar spine. At the same time, spiral CT has been widely used in clinical practice, making the scanning speed faster and faster and greatly expanding the scope of use. Therefore, this article combines spiral CT three-dimensional reconstruction to explore its clinical value in the diagnosis of lumbar degenerative osteoporosis.

At present, many experts and scholars have conducted research on the application of spiral CT three-dimensional reconstruction technology in the medical field and have obtained quite a wealth of research results. For example, Li et al. pointed out that spiral CT three-dimensional reconstruction imaging can comprehensively, carefully, and intuitively describe Crohn's disease intestinal wall thickening, intestinal pathology, and extraintestinal complications, which has an important guiding role in later clinical treatment [1]. Wang et al. explored the clinical value of three-dimensional multilayer spiral reconstruction in the diagnosis of female pelvic fractures and believed that the use of three-dimensional multilayer spiral reconstruction to examine patients with suspected pelvic fractures can help improve the diagnosis and provide a valuable evidence basis for imaging [2]. Ling believes that the use of CT three-dimensional reconstruction technology for thin-layer three-dimensional reconstruction of knee joint meniscus injury can show the information of meniscus injury to a greater extent and provide certain guidance for subsequent clinical diagnosis and treatment programs [3]. Therefore, from a new perspective, this article explores its clinical value in the diagnosis of lumbar degenerative osteoporosis in combination with the technical means of spiral CT three-dimensional reconstruction, which has important practical significance and research value to a certain extent.

This document deals mainly with these aspects. Firstly, it describes the three-dimensional reconstruction of the spinal cord and its research. This document introduces the concept and relevant investigation of vertebral degenerative osteoporosis. In addition, the implementation of the three-dimensional reconstruction of spiroid CT in the diagnosis of spinal degenerative osteoporosis was also discussed. Finally, in order to better understand the clinical value of the three-dimensional reconstruction of spiroid CT in the diagnosis of lumbar degenerative osteoporosis, this document has carried out an experimental survey and has obtained relevant experimental results and analytical conclusions.

RETRACTED

Through the research results of this paper, we can know that the image definition and accuracy of lumbar lesion location after three-dimensional reconstruction are high. Spiral CT three-dimensional reconstruction has an important clinical value in the diagnosis and treatment of lumbar degenerative osteoporosis. It is helpful to promote the diagnosis of three-dimensional reconstruction in lumbar osteoporosis.

## 2. Related Theoretical Overview and Research

### 2.1. Three-Dimensional Reconstruction of Spiral CT and Related Research

In recent years, the emergence of three-dimensional medical imaging has fundamentally changed the way of diagnosis and treatment and has become an indispensable and important means of clinical diagnosis and treatment. Three-dimensional medical images are more intuitive and accurate. With the help of computer graphics, different tissues can be displayed systematically and perfectly in three-dimensional reconstruction. At the same time, it also allows doctors to better locate the lesion and provide a certain degree of scientific basis to diagnosis and treatment for subsequent diseases.

Three-dimensional reconstruction of medical images is the application of computer graphics and image processing in biomedical engineering, and it is a multidisciplinary research field.

From the current point of view, the three-dimensional reconstruction methods of spiral CT mainly include surface rendering and volume rendering. Surface rendering is to extract the edges or contour lines of a two-dimensional image and then use geometric units to splice and fit the surface of the object to describe the three-dimensional structure of the object. Volume rendering is the direct application of vision principles to project voxels to a plane for display.

At present, there is no clear statement on the prediction of the location and size of blood or internal bone damage at home and abroad. When the three-dimensional reconstruction technology of multislice spiral CT is more and more used in the medical field, it brings a glimmer of hope for quickly solving this problem. Since the advent of spiral CT tomography, various image postprocessing technologies and corresponding computer tomography software have also been continuously improved, which greatly improves the quality and imaging speed of CT images [4, 5].

In addition, the multislice spiral computed tomography scan accurately provides a comprehensive visual view of the normal structure of the human body and the abnormal structure after the operation. The diagnosis of postoperative hematoma is also very clear, which can determine the source of hematoma, whether it is active bleeding and unit bleeding. If the bleeding does not stop within a short period of time, emergency surgery should be performed to stop the bleeding to avoid bleeding and cause the patient to die of unexplained hemorrhagic shock.

RETRACTED

It should be pointed out that the combination of 3D reconstruction and rapid prototyping (RP) technology provides an effective means for the design and manufacture of personalized implants. The use of three-dimensional images to design prostheses and rapid prototyping technology can meet individual needs. Using three-dimensional image to design prosthesis and rapid prototyping technology can meet personal needs and meet the characteristics of diversity, complexity and speed of prosthesis manufacturing.

Spiral CT became commercially available at the turn of the century, expanding its traditional ability to scan entire organs during a free diving cycle. The spiral brings the layer-oriented imaging process into the organ-oriented imaging process.

Spiral computed tomography data information is stored on the optical disc in accordance with digital medical imaging and communication standards, which can help operators to transmit and exchange digital images between medical imaging equipment more efficiently.

At present, medical imaging workstations such as CT and MRI all use 3D volume reconstruction, and this 3D reconstruction model cannot be directly used for engineering processing. Therefore, a computer is needed to process the spiral computed tomography data information stored on the optical disc.

Compared with conventional helix, three-dimensional helix has the following advantages.

Firstly, because the time between two scans of three-dimensional spiral is significantly shortened, the scanning of the whole organ can be completed in one respiratory cycle, and when more series are used, the scanning time is faster, and the reconstruction of cardiac scanning has no great impact on human heart rate.

Secondly, because the detection table moves at a uniform speed, it can be determined that the spiral scanning density direction is consistent, so the image can be reconstructed at any position. It can not only effectively reduce part of the volume effect but also facilitate postprocessing.

Third, nonoverlapping scanning can be used to create “overlapping images.” “Overlapping images” means that the distance between the reconstructed images is less than the thickness of the slice. The main advantage of reconstructing superimposed images is to produce reconstructed images [6, 7]. The image results of spiral CT three-dimensional reconstruction to check rib fractures are shown in Figure 1.

RETRACTED

A single-layer spiral sweep is similar to a fan sweep. The difference is that its projection has a fixed offset in the *z*-direction. Just add a *z*-direction offset to the projection sector formula for each projection angle. The spacing is defined as the ratio of the distance moved by the inspection table after the frame rotates one circle to the collimating aperture. The principle of single-layer spiral scanning can be expressed by

(1) $$\begin{array}{c} Q=\frac{a}{R}. \end{array}$$

Among them, *Q* is the pitch, *a* is the moving distance of the examination bed in one revolution of the frame, and *R* is the diameter of the collimator. If other parameters remain the same, if the spacing is too large, the gap between samples will change.

In spiral computed tomography, the data is continuously collected with the patient's body movement and the rotation of the scanner. Therefore, an interpolation method is needed to calculate the biological data of a specific slice of the patient and then reconstruct it. Commonly used interpolation methods are 180-degree and 360-degree interpolation.

The main difference between multislice spiral CT and single-slice spiral CT lies in the fundamental improvement of the detector design and data acquisition system. At the same time, it is also necessary to optimize the reconstruction algorithm and update related concepts. Regardless of the structure of the detector, the thickness of the scanning section can be determined by various combinations. Both symmetrical and asymmetrical detector designs have their own characteristics, and each has their advantages and disadvantages [8, 9].

Compared with single-layer spiral, multilayer spiral scanning is similar to cone-beam scanning, and the most commonly used techniques include optimized scan scanning and filter interpolation. The difference is that the projection of each angle has a fixed offset in the *z*-direction. As long as the simulation formula of cone beam scanning is added, every projection angle in the *z*-direction will produce a certain degree of cheapness. Different from the single-layer spiral sector sweep, the offset of the multilayer spiral in the *z*-direction can also be expressed by the pitch, but the definition of the pitch is changed. The principle of multilayer spiral scanning can be expressed by

(2) $$\begin{array}{c} Q=\frac{a}{n\cdot R}. \end{array}$$

Among them, *Q* is the pitch, *a* is the moving distance of the examination bed in one revolution of the frame, *n* is the number of detector rows, and *R* is the diameter of the collimator.

RETRACTED

### 2.2. Lumbar Degenerative Osteoporosis

At present, with the aging of the population, there are more and more degenerative diseases of the lumbar spine that accompany osteoporosis, and degenerative lumbar spine osteoporosis has also become fragile and high-incidence. This has also attracted the attention of scientists and experts in the medical field and other related fields.

Studies have shown that degeneration of the lumbar spine is an important factor in causing osteoporosis. At the same time, a vertebral fracture can increase the risk of vertebral fracture recurrence by 5 to 12.6 times, and the risk of hip fracture by 2.3 to 3.4 times. Approximately 20% of women with a single vertebra fracture will have a vertebral fracture again within a year. Multiply the risk of severe osteoporotic fractures by 4 and the risk of multiple vertebral fractures by 3. Spinal fractures can cause back pain, physical deformities, loss of social skills, decreased quality of life, and increased disability and mortality. In addition, it may also cause low back pain and radiation pain in the lower extremities. The occurrence of these complications will seriously affect the patient's quality of life.

There are many treatment methods for lumbar degenerative diseases. The use of pedicle screw internal fixation system for intervertebral fusion is the most widely used treatment method, which can effectively fix the segment, increase the stability of the intervertebral fusion, and reduce lumbar spine movement, thereby effectively reducing the occurrence of complications after fusion.

Lumbar degenerative disease is the general term for a series of conditions in which patients experience low back pain. In lumbar degenerative diseases, including mechanical pain and tenderness caused by degenerative changes of articular cartilage, lumbar intervertebral disc and ligaments around facets [10, 11]. Under normal circumstances, the degeneration of the lumbar spine is shown in Figure 2.

Advances in imaging continue to increase the diagnostic rate of degenerative lumbar spine diseases and at the same time significantly improve the accuracy of surgical positioning and reduce unnecessary blind exploration of the spinal canal during the operation.

The morphological structure of the vertebral body is the basis of the biomechanics of the vertebral body. The biomechanical changes caused by the degeneration of the intervertebral disc obviously affect the biomechanical structure of the vertebral body, and the changes in the internal structure of the vertebral body affect the overall shape and internal structure of the vertebral body. This has a very strong effect. The degeneration of the intervertebral disc can be accompanied by the degeneration of the vertebral body.

RETRACTED

In the process of lumbar joint degeneration, the shape of the joint can be reshaped, resulting in asymmetry of the small joints on both sides. Osteoporosis is a systemic bone disease that may have many causes. It is mainly manifested as the destruction of microstructure and the increase of bone fragility. The test can show bone density and bone loss. With the increase in the elderly population in my country, the prevalence of senile osteoporosis is significantly higher than in the past. Among the fractures of various parts caused by osteoporosis, vertebral body fractures and femoral neck fractures are the most common and early fractures, which are not uncommon in a clinical work. The incidence of vertebral fractures in white women over 50 years old is very high, and it gradually increases with age.

Under normal physiological conditions, the center of lumbar spine activity is behind the intervertebral disc. After the collapse, the pivot point retreats. If the degradation is severe, the pivot point can move to the facet joint. As the load on the facet joints increases, the shearing force with the lumbar spine increases, and the frictional force on the articular surface increases. This can initially manifest as an uneven cartilage on the joint surface and then develop into cartilage exfoliation and release of articular cartilage. The increase in mass density or osteomalacia will result in the growth of osteophytes on the edges of joints and bones and around the joints.

Degeneration of the lumbar spine can cause related clinical symptoms, such as low back pain, numbness of the limbs, and other clinical symptoms, which increase the probability of positive follow-up medical tests.

Osteoporosis is a common systemic bone disease in the elderly, and it has become a health problem of widespread concern. The clinical manifestations of osteoporosis mainly include frequent bone pain in the waist and hip and respiratory dysfunction, such as decreased vital capacity. The incidence of osteoporosis is gradually increasing. At present, the treatment of osteoporotic vertebral compression fractures with minimally invasive treatment technology has been widely recognized by the industry. The patient will benefit the most when the surgery involves only freshly compressed fractured vertebrae. Because patients with osteoporotic compression fractures often have multiple vertebral fractures and the old and new vertebral fractures alternate, it is often difficult to diagnose the vertebral body from the clinical symptoms.

RETRACTED

After a person suffers from osteoporosis, the bone density decreases and it is easy to cause fractures. Therefore, strengthening the treatment of osteoporosis, increasing bone density, and improving bone quality are of great significance for reducing the occurrence of fractures [10, 11].

### 2.3. Application of Spiral CT Three-Dimensional Reconstruction in the Diagnosis of Lumbar Degenerative Osteoporosis

The three-dimensional reconstruction of spiral CT is a milestone invention for neurosurgery. The wide application of spiral CT in clinic has greatly promoted the development of neurosurgery. In addition, the scanning speed is getting faster and faster, the scope of use is further expanded, and there is a wider space for the diagnosis of diseases.

At present, the most widely used clinical examination method is still X-ray imaging technology, which has the advantages of convenience and speed, but it cannot distinguish and diagnose new and old vertebral fractures.

The diagnosis of the vertebral body is based on imaging examinations. CT is widely used in clinical practice. It can show the structural changes in the vertebral body. Sometimes it can provide reliable imaging marks, such as clear fracture lines. It can identify and diagnose certain vertebral fractures. In addition, MRI has high sensitivity for the visualization of vertebral edema and is currently the main method to identify vertebral fractures.

Three-dimensional spiral CT reconstruction can combine bone metabolism with morphological images and has high differential diagnosis value. Three-dimensional spiral CT reconstruction is mainly used for the differential diagnosis of pathological vertebral fractures, and it also has a certain diagnostic value for bone mineral density and lumbar fractures. In short, imaging examination occupies an important position in the differential diagnosis of osteoporotic vertebral compression fractures.

With the widespread use of multislice spiral computed tomography, based on further examination of the disease and conventional sagittal reconstruction, many fractures have been found in patients. Compared with X-ray film, CT can observe the fine focus of fracture, which significantly improves the detection rate of fractured vertebrae. Because CT scans can show bones better than X-rays, it can better identify cortical injuries and injuries to the back of the spine.

For some occult fractures that cannot be detected by X-rays, CT can show the fracture line. If the edge of the fracture line is sharp or fuzzy, with freshness and age, the edge of the fracture line can be clearly seen. Fractures can be seen and need to be judged in advance. At the same time, three-dimensional reconstruction and thin-layer scanning technology have been widely used in a clinical work. The lesion can be observed at a free angle and in a free direction, whether the bone space structure is normal; whether the joint is dislocated, the number and boundary of the fracture, the type of fracture, and the end stage can clearly show the dislocation, soft tissue density, and morphological changes; and whether there are small fracture fragments. In addition, it performs CT examination in a clinical work and often detects other complicated diseases of patients, such as rib fractures, other old fractures, poor healing, osteoarthritis, and osteoporosis [12].

RETRACTED

This technology can clearly display the anatomical structure of the lumbar spine in the coronal, sagittal, and transverse positions and accurately measure the anatomy and separation area of the preperitoneal space required for osteoporosis, which provides a reliable suggestions and technical assistance for the subsequent treatment of the disease.

Three-dimensional spiral CT reconstruction is the most representative imaging examination in nuclear medicine. Whole body bone scan and bone tomography have been widely used in clinical practice and are most commonly used for the screening and diagnosis of tumor bone metastasis. A large number of studies have shown that on the basis of whole body bone imaging, the three-dimensional spiral CT reconstruction cofusion imaging combines CT imaging, which makes up for the shortcomings of bone metabolism imaging alone, and provides a wealth of imaging and bone metabolism information. It is very meaningful for the diagnosis of bone disease. In recent years, three-dimensional spiral CT reconstruction not only is used for the diagnosis of tumor bone metastasis but also has been paid more and more attention to its application in bone benign lesions. It has applied 3D spiral CT reconstruction to sports medicine research in forensic identification, sports medicine, and clinical and scientific research, such as fatigue fractures of ankles and calves, because many fatigue fractures have no changes in bone morphology. It is an occult fracture with slight edema, and neither CT nor MRI can be effectively diagnosed. The three-dimensional spiral CT reconstruction technique has high sensitivity and can effectively detect this part of the lesion. Some domestic studies believe that SPECT/CT and MRI have the same diagnostic efficacy in vertebral osteoporotic compression fractures and can be used as an alternative to MRI patients with contraindications. At the same time, three-dimensional spiral CT reconstruction technology can improve the operation of vertebral fractures. There is accuracy of segment positioning [13].

RETRACTED

## 3. Experiment and Research

### 3.1. Experimental Environment

In this experiment, the MX16-slice multislice spiral CT scanner was used. Scanning parameters are as follows: tube voltage is 160 V, tube current is 400-760 mA, layer thickness is 6 mm, layer spacing is 8 mm, spiral ratio is 1.375 : 1, and rotation speed is 0.7 s/r. The pitch is 0.984 : 1. After the scanning is completed, the thin layer is postprocessed and reconstructed. The thickness of the reconstructed layer is 0.85 mm, and the field of view is 20-55 cm.

### 3.2. Experimental Process

In this experiment, selected patients were initially diagnosed with degenerative osteoporosis of the lumbar spine and underwent imaging examinations in the Central Hospital of City A. The basic conditions of the patients are shown in Table 1. In this experiment, in order to understand the image results after three-dimensional reconstruction, five groups of cases were selected for testing. The test items include the overall lesion location, vertebral imaging, soft tissue lesion location, and lumbar lesion location. In addition, in order to understand the clinical value of spiral CT three-dimensional reconstruction technology in the diagnosis of lumbar degenerative osteoporosis, this technology and other imaging methods are compared and tested. The imaging methods selected for the experiment include X-ray, CT, and MRI. The test items include sensitivity, accuracy, positive predictive value, and negative predictive value.

## 4. Analysis and Discussion

### 4.1. Analysis of 3D Reconstruction Image Results

In this experiment, in order to understand the image results after three-dimensional reconstruction, five groups of cases were selected for testing. The test items include the overall lesion location, vertebral imaging, soft tissue lesion location, and lumbar lesion location. The experimental results are shown in Table 2.

It can be seen from Figure 3 that after the three-dimensional reconstruction, the clarity and accuracy of the relevant images of the five groups of cases are high; especially, the image reconstruction quality of the fifth group of cases is the highest, and the overall lesion location and vertebral imaging of the fifth group of cases, the sharpness and accuracy of the images, soft tissue lesion location, and lumbar lesion location were 0.97, 0.96, 0.95, 0.92, and 0.95, respectively. It can be obtained that the image quality of the image after the three-dimensional reconstruction is good, and the sharpness and accuracy are both high.

### 4.2. Comparison of the Clinical Value of Spiral CT Three-Dimensional Reconstruction Technology and Other Imaging Methods in Diagnosis

In this experiment, in order to understand the clinical value of spiral CT three-dimensional reconstruction technology in the diagnosis of lumbar degenerative osteoporosis, this technology and other imaging methods were compared and tested. The imaging methods selected for the experiment include X-ray, CT, and MRI. The test items include sensitivity, accuracy, positive predictive value, and negative predictive value. The experimental results are shown in Table 3.

RETRACTED

As shown in Figure 4, the sensitivity of X-ray, CT, MRI, and spiral CT 3D reconstruction is 85.3%, 87.3%, 87.1%, and 88.9%, and the accuracy is 90.1%, 89.4%, 93.6%, and 94.1%, respectively. It can be seen that the sensitivity and accuracy of spiral CT 3D reconstruction are higher than those of other imaging methods, and it has greater clinical value in the diagnosis and treatment of lumbar degenerative osteoporosis.

## 5. Conclusion

With the development of medicine, osteoporosis has been paid more and more attention. However, due to the complex and diverse internal structure of the human body and the interaction of various parts, it is difficult for patients to diagnose and treat, and it is easy to bring more pain to patients in the examination stage. In this case, spiral CT 3D reconstruction can give full play to its advantages. It has the advantages of simplicity, rapidity, and strong three-dimensional. It can clearly show the condition of lesions. Through the experimental study, it is found that after three-dimensional reconstruction, the relevant images of the five groups of cases have high definition and accuracy. The sensitivity and accuracy of spiral CT three-dimensional reconstruction are higher than those of other imaging methods. It has great clinical value in the diagnosis and treatment of lumbar degenerative osteoporosis. Therefore, in the clinical treatment of lumbar degenerative osteoporosis, three-dimensional reconstruction of patients with lumbar disease is very necessary. This paper concludes that the image definition and accuracy of lumbar lesion location after three-dimensional reconstruction are high, and three-dimensional spiral CT reconstruction has important clinical value in the diagnosis and treatment of lumbar degenerative osteoporosis.

## Figures and Tables

**Figure 1:** Spiral CT three-dimensional reconstruction of the image results of rib fractures.

**Figure 2:** Degeneration of the lumbar spine under normal circumstances.

**Figure 3:** Analysis of 3D reconstruction image results.

**Figure 4:** Diagnosis results of various imaging methods.

**Table 1:** The basic situation of the patients.

Age	Female	Male	Medical history	Spiral CT 3D reconstruction
40-50	0.1	0.08	0.05	0.37
51-60	0.22	0.2	0.18	0.36
61-70	0.25	0.29	0.22	0.24
71-80	0.32	0.33	0.3	0.27
Above 80	0.11	0.1	0.25	0.39

RETRACTED

**Table 2:** Analysis of 3D reconstruction image results.

Project	Group 1	Group 2	Group 3	Group 4	Group 5
Overall lesion location	0.93	0.91	0.96	0.94	0.97
Vertebral imaging	0.89	0.96	0.93	0.95	0.96
Location of soft tissue lesions	0.94	0.86	0.92	0.87	0.94
Lumbar lesion location	0.91	0.88	0.95	0.92	0.95

**Table 3:** Diagnosis results of various imaging methods.

Project	X-ray	CT	MRI	Spiral CT 3D reconstruction
Sensitivity (%)	85.3	87.3	87.1	88.9
Accuracy rate (%)	90.1	89.4	93.6	94.1
Positive predictive value (%)	83.4	86.7	88.4	89.1
Negative predictive value (%)	85.6	86.9	89.7	90.3

## Data Availability

The data underlying the results presented in the study are available within the manuscript.
